# K-ras-ERK1/2 down-regulates H2A.X^Y142ph^ through WSTF to promote the progress of gastric cancer

This article has been retracted.

**DOI:** 10.1186/s12885-019-5750-x

**Published:** 2019-05-31

**Authors:** Chao Dong, Jing Sun, Sha Ma, Guoying Zhang

**Affiliations:** 1 Department of Clinical Medicine, Qujing Medical College, Qujing, 655000 Yunnan China; 2 Department of Pharmacy, Qujing Medical College, Sanjiang Avenue, Economic Development Zone, Qilin District, Qujing, 655000 Yunnan China

**Keywords:** Gastric cancer, Ras-ERK, H2A.X^Y142ph^, WSTF, EYA3, MDM2

## Abstract

**Background:**

Histone H2AX phosphorylation at the site of Tyr-142 can participates in multiple biological progressions, which is including DNA repair. Ras pathway is closely involved in human cancers. Our study investigated the effects of Ras pathway via regulating H2AX.^Y142ph^.

**Methods:**

Gastric cancer cell line SNU-16 and MKN1 cells were transfected with Ras for G12D and T35S site mutation. The phosphorylation of H2A.X^Y142^ and ERK1/2, WSTF and MDM2 was detected by western blot. Cell viability, cell colonies and migration was analyzed by MTT assay, soft-agar colony formation assay, and Transwell assay, respectively. The expression of Ras pathway related downstream factors, EYA3 and WSTF was detected by qRT-PCR. The relationship between Ras and downstream factors were detected by ChIP. The cell cycle progression was measured by flow cytometry.

**Results:**

Ras^G12D/T35V^ transection decreased the phosphorylation of H2A.X^Y142^ and activated phosphorylation of ERK-1/2. H2A.X^Y142^ inhibited cell viability, colonies and migration. H2A.X^Y142ph^ altered the expression of Ras downstream factors. CHIP assay revealed that Ras^G12D/T35V^ could bind to the promoters of these Ras pathway downstream factors. Silence of EYA3 increased H2A.X^Y142ph^ and inhibited cell viability, migration and percent cells in S stage. Furthermore, silence of EYA3 also changed the downstream factors expression. WSTF and H2A.X^Y142ph^ revealed the similar trend and MDM2 on the opposite.

**Conclusion:**

Ras/ERK signal pathway decreased H2A.X^Y142ph^ and promoted cell growth and metastasis. This Ras regulation process was down-regulated by the cascade of MDM2-WSTF-EYA3 to decrease H2A.X^Y142ph^ in SNU-16 cells.

## Highlights

1. H2A.X^Y142ph^ is down-regulated by K-Ras-ERK1/2 in SNU-16 cells;
2. H2A.X^Y142ph^ restrains SNU-16 cell growth;
3. H2A.X^Y142ph^ down-regulates Ras downstream factors;
4. Silence of EYA3 up-regulates H2A.X^Y142ph^;
5. Ras-ERK1/2 induces WSTF degradation to down-regulate H2A.X^Y142ph^;
6. Ras-ERK1/2 down-regulates WSTF via MDM2.

## Backgroud

Increasing evidence suggests that abnormal Ras pathway is closely related with the progress of human cancer, but the exact epigenetic regulation mechanism is not clear [1, 2]. K-RasG12 is an oncogenic gene which is widely observed in human cancers [3]. In addition, the main downstream factors of Ras signaling included extracellular regulated protein kinases (ERK) 1/2, phosphatidylinositol 3′-kinase (PI3K), and Ras-like (Ral) 2 guanine nucleotide exchange factors (RalGEFs) [4–6]. However, the detailed information and the underlying mechanisms how Ras signal pathways involved are still not well understood and studied.

It is well-known that eukaryotic DNA is wrapped by histone octamers which was made of four different kinds of histones, H2A, H2B, H3 and H4. Importantly, the post-transcriptionally modification of histone N-terminal tail can regulate chromatin organization and DNA utilization processes, including transcription [7]. With the development of science and technology, the deciphering of histone code and its biological functions has received increasing attention. A substantial amount of studies point out that histone modification is subjected to a wide range of tumor [8]. For example, a study from Yang et al. found that histone modification is involved in regulating tumorigenesis of gastric cancer (GC) [9]. The silencing or removing H2A.X, a histone variant, was involved in cellular DNA repair and robust growth [10]. Interestingly, the roles of histone modification received considerable attention in GC [11]. For example, hypoxia silences runt-related transcription factor 3 (RUNX3) by epigenetic histone modification in the progression of GC [12]. Histone deacetylases expression is an independent prognostic marker in GC [13]. These finding sindicated that histone modification exert paramount important role in GC.

H2A.X is the damage-related histone variant, which is identified by the C-terminal tyrosyl residue, Tyr-142. The reason for that is Tyr-142 could be phosphorylated by an atypical kinase, Williams-Beuren syndrome transcription factor (WSTF) and inducing phosphorylation of H2A.X into H2A.X^Y142ph^ [14, 15]. High level of Tyr142 phosphorylation regulates several biological progressions, including apoptosis and DNA repair [14]. Meanwhile, the effects of dephosphorylation for the eyes absent homolog (EYA) 1/3 also address novel insight into this process [16]. Therefore, we investigated the role of Ras-ERK pathway in cell viability, colonies and migration via the regulation of H2A.X^Y142ph^. Finally, we investigated the underlying mechanisms in gastric cancer cell line SNU-16 and MKN1 cells.

## Material and methods

### Cell culture

Human GC cell line SNU-16 and MKN1 cells were purchased from Shanghai Institute for Biological Science (Shanghai, China). Cells were maintained at 37 °C, 5% CO_2_ in RPMI-1640 (Gibco Laborato-ties, Grand Island, NY) with 100 units/ml penicillin, 100 μg/ml streptomycin and 10% fetal bovine serum (FBS, Life Science, UT, USA).

### Plasmid construction and siRNA

Empty-pEGFP-N1 vector, pEGFP-K-Ras^WT^, pEGFP-K-Ras^G12V/T35S^ plasmids were transfected in cells. The transfection with specific gene with HA-tag was used for screening out the target factor through western blot. pEGFP-K-Ras^G12V/T35S^ plasmids were obtained by site-directed mutagenesis. SiRNAs (Shanghai GenePharma, Shanghai, China) refers to using interference RNA to silence the goal RNA (Mouse double minute 2 homolog (MDM2) or EYA3). The pEGFP-H2A.X^Y142A^ construct was constructed using the TaKaRa MutanBEST Kit (#D401) (TaKaRa, Shiga, Japan) as recommend by the manufacturer.

### Transfection

Cells at the density of 5 × 10^5^ per well were cultured in 6-well plates for 12 h in the darkness. Then the cells were transfected with plasmids or siRNA using Lipofectamine 2000 (Invitrogen, Carlsbad, CA). Then qRT-PCR and western blot were used to determine the transfection efficiency after 48 h of transfection.

### Cell viability

MTT (Sigma-Aldrich, St Louis, MO, USA) was used for the detecting cell viability. After cells were cultured for 48 h, 20 μl 5 mg/mL MTT was administrated to each well. Cells were cultured for 4 h. Afterward, we used 100 μl dimethyl sulfoxide (Sigma-Aldrich, St Louis, MO, USA) to lyse formazan crystal. The value was obtained at 570 nm by a multiwell spectrophotometer (Emax; Molecular Devices, Sunnyvale, CA).

### Reverse transcription polymerase chain reaction (RT-PCR)

RT-PCR method was referred to what described in the report [17]. Total RNA was obtained from SNU-16 cells using TRIzol (Invitrogen) reagent. DNase-I-treated total RNA was supplied for first-strand cDNA synthesis by M-MuLV reverse transcriptase (Fermentas, York, UK) and oligo-dT primers (Invitrogen). QuantiTect SYBR Green PCR Kit (Qiagen, Hilden, Germany) was used to amplify the target sequence. GAPDH was an internal control for detecting RNA expression based on triplicate experiments.

### Soft-agar colony formation assay

Soft-agar assay was performed to measure the cell colonies ability [18]. The cells suspended in full culture medium with 0.35% low-melting agarose, then cells were transferred into solidified 0.6% agarose in six-well culture plates (1 × 10^3^ cells/well). The number of the colonies was counted 3 weeks later using microscopically (40 ×).

### Transwell migration assay

Cell migration was evaluated by using a modified two-chamber migration Transwell (Corning Costa, NY, US) with a pore size of 8 μm. 100 μl (around 2 × 10^5^ cells/ml) cell suspension without serum was added to upper Transwell. 600 μl complete medium was added in the lower compartment. Cells were maintained for 24 h at 37 °C, 5% CO_2_. After incubation, cells at the upper surface of the filter were removed by a cotton swab, and the filter was fixed with methanol for 5 min. Cells at the lower surface of the filter were stained by 0.1% Giemsa (Sigma-Aldrich) for 15 min. Cells were counted by 100 × microscope.

### Western blot analysis

Protein was obtained using RIPA lysis buffer (Cat. No:R0010, Solarbio, Beijing, China) supplemented with protease inhibitors (Thermo Fisher Scientific, Rockford, IL). The BCA™ Protein Assay Kit (Pierce, Appleton, WI, USA) was used for determining protein concentrations. Western blot system was established using a Bio-Rad Bis-Tris Gel system following the manufacturer’s instructions. Primary antibodies were prepared in 5% blocking buffer and diluted according to the product instruction. These primary antibodies were incubated in membrane and maintained at 4 °C overnight at recommended concentration. Then secondary antibody incubated with horseradish peroxidase (HRP) conjugated secondary antibody. Captured the signals, and Image Lab™ Software (Bio-Rad, Shanghai, China) quantified the intensity of the bands.

### Flow cytometric analysis of cell cycle distribution

SNU-16 cells were cultured until reach 75–80% confluence, and then cells were washed by PBS to remove the non-adherent cells. Collected cells were all adherent cells and fixed with cold 70% ethanol. Cells were washed with PBS again. After that, cells were stained with 4, 6-diamidino-2-phenylindole (DAPI) (Partec, Germany) and cultured in the darkness for 30 min. Flow cytometry was used for detecting cell cycle distribution. The percentage of cells in different cell cycle stages was calculated.

### Chromatin immunoprecipitation (ChIP)

Cells were fixed in 1% formaldehyde, then lysed, and sonicated cells. Then 5 mg chromatin was immunoprecipitated with Dynabeads. After that, purified DNA was used for PCR amplification at the CYR61, IGFBP3, WNT16B, NT5E, GDF15, CARD16 promoter. The detailed process could refer to the literature [19].

### Statistical analysis

Data was analyzed by Graphpad 6.0 statistical software (GraphPad, San Diego, CA, USA). Data were present as mean + SD. The statistical analyses were performed using the Student’s t-test or one way ANOVA followed by *Duncan post-hoc* of multiple comparisons. A *P* value of < 0.05 was considered significant (* *P* < 0.05, ** *P* < 0.01 or ***P < 0.001).

## Results

### H2A.X^Y142ph^ was down-regulated by Ras-ERK1/2 pathway

Ras/ERK signal pathway was often found to be closely related with GC [20]. In our study, SNU-16 and MKN1 cells were respectivly transfected with empty-pEGFP-N1 vector, pEGFP-K-Ras^WT^ and pEGFP-K-Ras^G12V/T35S^ plasmids. Results showed that Ras^G12V/T35S^ decreased the expression of H2A.X^Y142ph^ level (*P* < 0.01, Fig. 1a). In addition, we measured the effects of Ras^G12V/T35S^ activated phosphorylation of ERK1/2 (Fig. 1b). To confirm this suggestion, another cell line MKN1 was used and similar results were also observed in this cell line as what we describe in SNU-16 cells (*P* < 0.01, Fig. 1c-d), which suggested that Ras^G12V/T35S^ played a role as a switch for the phosphorylation of ERK.

**Fig. 1:** H2A.X^Y142ph^ was down-regulated by Ras-ERK1/2 pathway. SNU-16 cells and MKN1 cells were transfected with empty-pEGFP-N1 (pEGFP-N1), pEGFP-K-Ras^WT^ (Ras^WT^), pEGFP-K-Ras^G12V/T35S^ (Ras^G12V/T35S^) plasmids. **a** The H2A.X ^Y142ph^ levels and (**b**) the phosphorylation of ERK1/2 were measured using western blot in SNU-16 cells. **c** The H2A.X ^Y142ph^ levels and (**d**) the phosphorylation of ERK1/2 were measured using western blot in MKN1 cells. Data presented as mean + SD, ** *P* < 0.01 (*n* = 3)

### H2A.X^Y142ph^ restrained Ras pathway on GC cell phenotype

Histone modification influenced cell growth and cell metastasis [21]. In the current study, we constructed H2A.X^Y142A^ plasmids to mimic the situation of the phosphorylation of H2A.X^Y142^. The mimicked H2A.X^Y142A^ plasmids were co-transfected with Ras^G12V/T35S^ plasmids into SNU-16 cells and MKN1 cells. Hence, we examined the effects of phosphorylation of histone H2A in GC cell viability, cell colony ability and cell migration. Firstly, SNU-16 cell was transfected with H2A.X^Y142A^.With the increasing concentration, the expression of phosphorylation of H2A.X^Y142^ was inhibited in a dose-dependent manner (Fig. 2a). Moreover, results showed that Ras/ERK pathway significantly increased cell viability (*P* < 0.001) while H2A.X^Y142A^ decreased cell viability to some extent in SNU-16 cells (*P* < 0.001, Fig. 2b). This result suggested that Ras/ERK has the ability to increase cell viability while H2A.X^Y142A^ decreased cell viability, which indicating H2A.XY142A suppressed cell growth in GC. In addition, the number of colonies (*P* < 0.01, Fig. 2c) and cell migration (*P* < 0.001, Fig. 2d) revealed the similar trend by Ras^G12V/T35S^ pathway in SNU-16 cells. Similar results were also observed in MKN1 cell line (*P* < 0.05 or *P* < 0.01, Fig. 2e-h). Taken together, we inferred that the phosphorylation of H2A.X^Y142^ was involved in the progression of GC cells.

**Fig. 2:** H2A.X ^Y142ph^ restrains SNU-16 cell growth. SNU-16 cells were transfected with pEGFP-N1, pEGFP-H2A.X, pEGFPH-Ras^G12V/T35S^, or pEGFP-H2A.X^Y142A^ (indicated as GFP, H2A.X, Ras^G12V/T35S^ and H2A.X ^Y142A^, respectively) plasmids. **a** The expression of H2A.X ^Y142ph^ levels were detected by western blot. **b** Cell viability, (**c**) numbers of colonies and (**d**) cell migration were detected by MTT assay, soft agar, and Transwell assays, respectively in SNU-16 cells. (**e**) The expression of H2A.X ^Y142ph^ levels were detected by western blot. **f** Cell viability, (**g**) numbers of colonies and (**h**) cell migration were detected by MTT assay, soft agar, and Transwell assays, respectively in MKN1 cells. Data presented as mean + SD, * *P* < 0.05, ** *P* < 0.01, *** *P* < 0.001 (*n* = 3)

### H2A.X^Y142ph^ down-regulated the downstream factors of Ras pathway

Ras/ERK pathway was a complex and exact regulation pathway which was modulated by diverse downstream factors [22]. We explored the expression of these important downstream factors CYR61 [23], IGFBP3 [24], WNT16B [25], NT5E [26], GDF15 [27], CARD16 [28], which are involved in the tumor cell growth and cell metastasis. Then, we found that Ras^G12V/T35S^ increased the expression of WNT16B (*P* < 0.05), NT5E (*P* < 0.01) while decreased the expression of IGFBP3 (*P* < 0.01), GDF15 (*P* < 0.01) and CARD16 (*P* < 0.01). Meanwhile, we found that co-transfection with Ras^G12V/T35S^ and H2A.X^Y142A^ decreased the expression of CYR61 (*P* < 0.05), IGFBP (*P* < 0.001), WNT16B (*P* < 0.05) and increased the expression of NT5E (*P* < 0.05), GDF15 (*P* < 0.05) and CARD16 (*P* < 0.05) as relative to Ras^G12V/T35S^ group, which suggested that H2A.X^Y142A^ was down-regulated these downstream genes of Ras^G12V/T35S^ pathway. In addition, the ChIP assay results showed Ras^G12V/T35S^ decreased expression of these genes (*P* < 0.05, *P* < 0.01 or *P* < 0.001, Fig. 3b), this suggested that H2A.X^Y142ph^ could down-regulate gene expression via directly binding to these gene’s promoters. In conclusion, H2A.X^Y142ph^ could down-regulate the downstream transcription progression of the downstream factors.

**Fig. 3:** H2A.X ^Y142ph^ down-regulated the downstream factors of Ras pathway. The transcription of Ras-ERK1/2-targeted genes can be partially down-regulated by increased H2A.X^Y142ph^. **a** The transcription of several genes was tested using real time PCR. **b** As detected using ChIP, reduced levels of H2A.X^Y142ph^ are present on the differentially expressed genes. Data presented as mean + SD, ns, no significant difference, * *P* < 0.05, ** *P* < 0.01, *** *P* < 0.001 (*n* = 3)

### Knockdown of EYA3 up-regulated H2A.X^Y142ph^ expression and recovered the GC cell phenotype

Previous study reported that the effects of dephosphorylation of histone H2A by the EYA1/3 also address significant influence in human cancers [16]. Thereafter, knock-down EYA3 expression to investigate whether upregulation of phosphorylation of H2A.X^Y142^ could modulate cell phenotype was performed. qRT-PCR and western blot was used to determine the transfection efficiency. We used two interference miRNAs to silence the expression of EYA3, which named si-EYA3–1 and EYA3–2, respectively. Result in Fig. 4a showed that si-EYA3–1 and si-EYA3–2 both decreased EYA3 expression in mRNA level and adding si-EYA3–1 and si-EYA3–2 both up-regulated the phosphorylation of H2A.X^Y142^. After that, we detected the effects of si-EYA3–1/2 on cell viability, cell migration, cell cycle stage and cell relative mRNA levels. Results showed that si-EYA3–1/2 decreased cell viability (*P* < 0.05), cell migration (*P* < 0.05) and cell percent in S stage as compared with Ras^G12V/T35S^ alone (Fig. 4b-d). Furthermore, EYA3–1/2 also altered the expression of the downstream factors of Ras^G12D/T35V^ pathway compared with Ras^G12V/T35S^ alone in GC cells (*P* < 0.05, *P* < 0.01 or *P* < 0.001, Fig. 4e), which suggesting that EYA3 also participated in the regulation of the downstream factors of Ras^G12V/T35S^ pathway.

**Fig. 4:** Silence of eyes absent homolog (EYA) 3 up-regulated H2A.X^Y142ph^. **a** The efficiency of siRNA-mediated EYA3 knockdown was determined. The depletion of EYA3 prevented the Ras-ERK1/2 activation-induced decrease in the H2A.X^Y142ph^. SNU-16 cells were co-transfected as indicated. Whole cell lysates were assayed using western blot. SNU-16 cells were co-transfected with pEGFP-K-RasG^12V/T35S^ or pEGFP-N1 plasmids and EYA3-specific or control siRNA as indicated (Ras, GFP, si-EYA3–1, si-EYA3–2, or si-con, respectively). **b** Cell viability, (**c**) cell migration, (**d**) cell cycle progression were detected by MTT assay, Transwell assays and flow cytometry, respectively. (**e**) Silence of EYA3 on downstream factors was detected by real time RCR. Data presented as mean + SD, * *P* < 0.05, ** *P* < 0.01, *** *P* < 0.001 (*n* = 3)

### Ras-ERK1/2 induced WSTF degradation to decrease H2A.X^Y142ph^ expression

WSTF makes mutant H2A.X phosphorylated in Tyr 142, and the activity of WSTF exert indispensable functions in regulating multiple events [29]. Further experiments were performed to explore the exact mechanism how WSTF affects the phosphorylation of H2A.X^Y142^. Result from Fig. 5a showed that no obviously difference was observed in the expression of WSTF and EYA3 in the group pEGFP-N1 and Ras^G12V/T35S^. This suggested that WSTF was not played part in the transcription level. Afterwards, we found that the expression of EYA3 in protein level was no difference (Fig. 5b) while WSTF was significantly decreased (Fig. 5c) in the group Ras^G12V/T35S^. Combined the result of Fig. 5b and c, we inferred that the effects of WSTF induced by Ras^G12V/T35S^ was in translation level. Interestingly, the result in Fig. 5d confirmed our inference, WSTF and H2A.X^Y142ph^ revealed the same trend reacted in group Ras^G12V/T35S^. Further result showed that Ras^G12V/T35S^ could bind to the promoters of genes to reduce the input levels of WSTF in downstream factors of Ras^G12V/T35S^ pathway (Fig. 5e). Moreover, the proteasome inhibitor MG132 administration made the changes of WSTF expression by Ras^G12V/T35S^ disappeared, which indicated high inhibition for WSTF (Fig. 5f). Afterwards, we found that without MG132 administration, the phosphorylation level of H2A.X^Y142ph^ was decreased with the delaying of the transfection time (24, 48, 51, 54 and 60 h) in SNU-16 cells (Fig. 5g). Similar, under the same treatment, we found that the accumulated levels of WSTF was decreasing with the increasing of the transfection time (Fig. 5h). On the opposite, with the MG132 supplement, the decreased phosphorylation level of H2A.X^Y142ph^ by Ras^G12V/T35S^ was vanished. Instead the phosphorylation level of H2A.X^Y142ph^ was increased after administration of MG132 in different time treatment (0, 3, 6 and 12 h) (Fig. 5i). Taken together, these findings indicated that Ras^G12V/T35S^ pathway affected the phosphorylation of H2A.X^Y142ph^ was through WSTF.

**Fig. 5:** Ras-ERK1/2 induced Williams–Beuren syndrome transcription factor (WSTF) to decrease H2A.X^Y142ph^. **a**-**d** SNU-16 cells were transfected with pEGFP-K-Ras^G12V/T35S^, pEGFP-N1, and WSTF-HA or EYA3-HA plasmids. 24 h later, RNA was collected and detected by PCR; 48 h later, cell lysates were analyzed using western blot. **e**The recruitment of WSTF to the genes that exhibited changes in H2A.X ^Y142ph^ was analyzed using ChIP analysis. **f** Whole cell extracts from SNU-16 cells that were treated with MG132 were prepared, and the WSTF protein levels were analyzed using western blot with antibodies against HA and GFP. **g**-**i** Whole cell extracts from SNU-16 cells that were untreated (the samples were collected at 24, 48, 51, 54, and 60 h following transfection; upper panel) or treated with MG132 (the MG132was added at 48 h following transfection, and the samples were collected at 24, 48, 51, 54, and 60 h following transfection; lower panel) were analyzed using western blot. Data presented as mean + SD, * *P* < 0.05, ** *P* < 0.01, *** *P* < 0.001 (*n* = 3)

### Ras-ERK1/2 down-regulated WSTF via MDM2

It is well validated that histone modification was mediated by MDM2 in various cells [30]. Further experiments were performed to explore the mechanism about whether MDM2 was involved in the regulation of WSTF on H2A.X^Y142ph^. We co-transfected Ras^G12V/T35S^ and WSTF with tagged HA into cells. The result of western blot showed that WSTF expression was decreased with the increasing of MDM2 (Fig. 6a). Further result showed without transfecting WSTF, the expression of WSTF was still decreased with the increasing of MDM2, which indicated that there might be a negative relationship between MDM2 and WSTF (Fig. 6b). Furthermore, we co-transfected Ras^G12V/T35S^ and WSTF with tag HA, the expression of WSTF was inhibited when transfected MDM2-His while WSTF expression was enhanced when transfected MDM2-MU (Fig. 6c), which strongly suggested that there was closely negative relationship between MDM2 and WSTF expression. Moreover, As shown in Fig. 6d, Ras^G12V/T35S^ and detected the expression of WSTF got the similar result as Fig. 6c, which confirmed the strong negative association between MDM2 and WSTF. We thereafter determined the relationship between MDM2 and H2A.X^Y142 ph^ and result in Fig. 6e. The result showed that Ras^G12V/T35S^ inhibited H2AX.^Y142ph^ while up-regulated MDM2 expression. Then si-MDM2 to silence MDM2 (Fig. 6f) and we found that si-MDM2 could enhance the expression of H2A.X^Y142ph^, which confirmed the result in Fig. 6e. Then through these experiments, we concluded the cascade reaction might be Ras^G12V/T35S^ positively regulated MDM2 expression, and then MDM2 negatively regulated WSTF, and WSTF positively regulate H2A.X^Y142 ph^.

**Fig. 6:** The Ras-ERK1/2 signaling pathway-induced degradation of Williams-Beuren syndrome transcription factor (WSTF) is mediated by mouse double minute 2 homolog (MDM2). **a**-**b** MDM2 induces the degradation of WSTF. SNU-16 cells were co-transfected with WSTF-HA, pEGFP-K-Ras^G12V/T35S^, of pEGFP-N1 plasmids and increasing amounts of MDM2-His plasmid (0.5, 1, and 2 g). **c**-**d** A mutation in MDM2 (MDM2-MU) that abolishes its ubiquitin ligase activity prevents WSTF degradation. The SNU-16 cells were co-transfected as indicated. **e** Whole cell extracts from SNU-16 cells that were transfected with pEGFP-N1 or pEGFP-K-Ras^G12V/T35S^ were analyzed using western blot. **f** The efficiency of the siRNA-mediated MDM2 knockdown. **g** The co-transfection of pEGFP-K-Ras^G12V/T35S^ and MDM2-specific siRNA restores H2A.X^Y142ph^ to normal levels

## Discussion

The alternation of epigenetic modifications might be a key reason in the progress of cancer, including gastric cancer [12]. Epigenetic modifications include diverse forms, such as the methylation of cytosines on DNA, and N-terminal of the histone proteins (H2A, H2B, H3 and H4). Importantly, because its main reason causing aberrant gene damage, histone modification which included acetylation, methylation, phosphorylation and ubiquitylation of the specific histones receives great attentions worldwide now. It also becomes a hallmark of human cancer progress [31]. In the other hand, it is well-known that Ras pathway is involved in diverse human cancers, such as colorectal cancer [32] and colon cancer [33]. Importantly, Ras/ERK is the effective approach in the regulation of cell proliferation and cell invasion in GC [34]. In our study, we investigated the effects of H2A.X^Y142ph^, Ras^G12V/T35S^ pathway and the underlying mechanisms in gastric cancer cell SNU16 and MKN1 cells.

H2A.X is the histone H2A family variant, and the H2AX C-terminal domain could be phosphorylated by tyrosine 142 by the WSTF remodeling factor kinase [29]. The expression of H2A.X^Y142ph^ was related to DNA damage. In our study, we found that site mutation of G12 V and T35S in Ras pathway decreased the expression of H2A.X^Y142ph^, which indicated that Ras^G12V/T35S^ might worked through down-regulated H2A.X^Y142ph^. In addition, further result also proved that Ras^G12V/T35S^ was a switch of phosphorylation of ERK1/2, which suggested that Ras/ERK might play a vital role in regulation of H2A.X^Y142ph^.

Cell viability, cell colonies and cell migration was three important factors for judging cell growth and cell metastasis. Ras/ERK signaling pathway was often found activated in multiple human cancers [35], we explored the effects of Ras on GC cells SNU-16 and MKN1 cells. In our study, experiments explored whether Ras^G12V/T35S^ and H2A.X^Y142ph^ worked in cell viability, number of colonies and cell migration. Result showed that Ras/ERK pathway could enhance cell viability, cell colonies and cell migration, this consistent with the previous studies that activation of ERK pathway promoted GC cell growth [36]. On the other hand, H2A.X^Y142ph^ reversed the results, which suggested that phosphorylation of H2A.X might regulate GC cell growth and metastasis. Meanwhile, histone modification exerts crucial functions in the progress of cancer. For example, pancreatic cancer cell growth and metastasis was modulated by histone modification of P27, P53 and Bax [21]. We therefore inferred that histone modification of H2A.X^Y142ph^ could affect cell growth might also through regulating the downstream related genes.

Next, results revealed that Ras/ERK down-regulated downstream factors, CYR61, IGFBP3, WNT16B, NT5E, GDF15 and CARD16. Meanwhile, phosphorylation of H2A.X exert the opposite functions as compared with Ras/ERK pathway, this suggested that phosphorylation of H2AX might play important role in modulating Ras/ERK pathway. CHIP assay result showed that Ras/ERK significantly decreased all the gene expression, which confirmed that H2A.X^Y142ph^ could up-regulated the downstream factors.

EYA phosphatases are responsible for the phosphorylation of H2A.X on the C-terminal of tyrosyl residue, and EYA2 and EYA3 were proved to be for specificity for Tyr-142 of H2A.X [15]. Results showed that silence of EYA3 increased H2A.X^Y142ph^, further results demonstrated that silence of EYA3 decreased cell viability, cell migration, the percentage of S stage and alter the downstream factors expression in RNA level. These result showed that downregulation of EYA3 led to enhancement of phosphorylation and reduced DNA-damage dephosphorylation of Tyr-142 of H2A.X in vivo [15]. These findings suggested that silence of EYA3 revealed the similar trend with H2A.X^Y142ph^.

In the beginning, we knew that H2A.X^Y142ph^ was phosphorylated by WSTF [14, 15]. Then we asked how WSTF was involved in the phosphorylation progress? After, we detected the role of WSTF in SNU-16 cells. We found that no different was found in the RNA level between Ras^G12V/T35S^ pathway with the control, which indicated that the effects of WSTF were not in the transcription level. Then we found that WSTF showed that similar trend under transfection with Ras, and further CHIP assay showed that Ras^G12V/T35S^ could bind to the promoters of genes to reduce the input levels of WSTF in downstream factors of Ras pathway. Further result showed that activity of Ras-ERK1/2 induced WSTF degradation to decrease H2A.X^Y142ph^ expression.

In the last, we studied the mechanism how WSTF was regulated in the progression. MDM2 displays important role in histone ubiquitylation and transcriptional repression [30]. Result demonstrated that Ras/ERK degraded WSTF through upregulation of MDM2. MDM2 revealed negative relationship with H2A.X^Y142ph^ expression. Taken together, the whole cascade process might be MDM2 negatively regulate WSTF, WSTF positively regulated EYA3, and EYA3 positively regulated H2A.X ^Y142ph^, which was down-regulated by Ras^G12V/T35S^.

## Conclusions

In conclusion, our result demonstrated the Ras^G12V/T35S^ and H2A.X^Y142ph^ in regulating GC cell growth. The underlying mechanisms are also explored. We firstly found that Ras/ERK pathway could promote GC cell growth while H2A.X^Y142ph^ inhibited cell growth. Our study proved the importance of histone modification to some extent. At the same time, we provided novel insight in the relationship between histone modification and the treatment of GC.

## Data Availability

The datasets used and analyzed during the current study are available from the corresponding author on reasonable request.

## Abbreviations

ChIP: Chromatin immunoprecipitation
ERK: Extracellular regulated protein kinases
FBS: Fetal bovine serum
GC: Ras-like (Ral), Gastric cancer
HRP: Horseradish peroxidase
PI3K: Phosphatidylinositol 3′-kinase
RT-PCR: Reverse transcription polymerase chain reaction
RUNX3: Runt-related transcription factor 3
WSTF: Williams-Beuren syndrome transcription factor
